# Evaluation Algorithm for Team Strength Based on the Collected Healthcare Data through IoT and Smart Devices

This article has been retracted.

**DOI:** 10.1155/2022/4969527

**Published:** 2022-01-07

**Authors:** Jian Qiao

**Affiliations:** Department of Fine Art, Music and Physical Education, Henan College of Transportation, Zhengzhou, 450000, China

## Abstract

In the past, the fans used to evaluate the strength of the team according to the victory and defeat ranking or according to their own intuition and preferences, however, the strength of the team is difficult to measure in analytical figures. The team's winning rate is not the only factor to be considered to determine the strength of the team. There are many factors to be considered for determining the strength of the team. According to the variation coefficient of basketball scoring frequency, the paper designs the principal model of basketball players' pitching target system. The data is captured by IoT devices and smart devices. The algorithm sets the number of the frequency of Gabor filter transformation features, controls the error accumulation, extracts the cascade features of basketball score video, constructs the video conversion discrimination rules, detects the basketball target, and obtains the tracking target contour to frame information. Finally, it realizes the target tracking detection of the team based on the team strength using an evaluation algorithm. The aim of this research work is to determine the strength of the team based on the healthcare data, team cohesiveness, and variance coefficient of basketball score frequency. The study on the coefficient of variation for basketball score frequency in teams can provide a theoretical research direction for team strength evaluation and meet the real-time needs of the coefficient of variation of basketball score frequency in teams. The empirical results show that the designed algorithm has the optimal execution time, more successful evaluation targets, high efficiency, and more reliability in evaluating the strength of the team.

## 1. Introduction

Because of the popularity and substantial commercial value of competitive sports, the internet has carried out data statistics on all kinds of basketball matches, given the performance of each team, and ranked the teams. The game followers often evaluate the strength of the group according to the victory and defeat ranking or divide the unity strength according to their own intuition and preferences [1–3]. However, because of the different logarithmic strength of the team that has competed and as the score difference between the winner and the loser of each competition has not been considered, the winning rate cannot correctly reflect the strength of the team. In the era of big data, we should make a scientific and reasonable evaluation based on the existing historical competition data. Therefore, it has certain research value and practical significance for team strength evaluation [4, 5].

There is research on team strength evaluation. Reference [6] proposes the scale and strength evaluation of the training team learning direction. It studies how the heterogeneity of team personality affects the size and strength of team learning, which is inspired by transformational leadership, behavior combinations, extroversion, and agreeability. Transformational leadership can gather high-intensity learning orientation in the work team by promoting behavior amalgamation among the team members. However, the influence of transformational leadership greatly depends on the degree of heterogeneity of personalities of the team members. Transformational leaders must foster the sharing of information among the players and participation in decision-making among team members to decide the cohesion of the team. Reference [7] suggested analyzing basketball players' movements and evaluating team effectiveness. It also examined the background information and indications utilized in advanced basketball to assess the team's strength. The benchmarked techniques along with the designed techniques are used to evaluate teams and players. There are many techniques in the literature proposed by the researchers to evaluate team strength [8].

Team characteristics analysis may be used to determine team composition and measure team strength for future forecasting. It can assist them better in understanding the game's benefits and drawbacks and helps get a better assessment of the other team. Performance indicators may also be improved, and these indications can help anticipate player behavior and team participation. Despite the fact that existing research has progressed, it is still impossible to determine the analysis of team scores. As a result, this study develops a team strength evaluation method based on the variation coefficient and draws a valid conclusion. The data is collected from the sportspersons from the Chinese sports academy. The data is based on the questionnaire, and the records are recorded using smart devices. The IoT-based smart devices are used to sense the person's opinion in a better manner and know whether the person is giving a true statement. Secondly, the performance of the players in the past from their experiences is also recorded using their healthcare data, such as perceived stress score, Epworth Sleepiness Scale, BPM (beat per minute), winning times, failure times, and improvement in time management. The need to collect healthcare-related data also contributes to the success and failures of the teams. If the players are stressed, then they cannot perform well. If the players do not sleep well, then they cannot perform well. Their overall physical and mental health plays a major role in deciding their success and failure in the games. It also impacts their overall performance.

### 1.1. Contributions of the Paper

- This paper proposes a team strength evaluation algorithm based on the variation coefficient of basketball scoring frequency.
- According to the variation coefficient of basketball scoring frequency, the paper designs the principle model of basketball players' pitching target system.
- The data is captured by IoT devices and smart devices. The algorithm sets the number of the frequency of Gabor filter transformation features, controls the error accumulation, extracts the cascade features of basketball score video, constructs the video conversion discrimination rules, detects the basketball target, and obtains the tracking target contour and frames information.
- Finally, it realizes the target tracking detection of the team based on the team strength using an evaluation algorithm.
- The evaluation of the team strength is made on the basis of the variation coefficient of basketball score frequency. The empirical results show that the designed algorithm has the shortest execution time, more successful evaluation targets, high efficiency, and more reliability in evaluating the strength of the team.

### 1.2. Structure of the Paper

Section 1 provides the introduction and contributions of the paper, along with a brief discussion of related work.  Section 2 showcases the methodology of the proposed work done in this paper. The analysis of experimental results is done in Section 3. A thorough discussion of the outcomes is done in Section 4, followed by the conclusion section and references.

## 2. Basketball Score Frequency Mutation Coefficient Team Strength Evaluation Algorithms

To apply the algorithms, it is very important to collect the data very carefully. Hence, the healthcare-based complex data is used in this research work to measure the performance of the players. The combination of physical and mental health makes the players strong. They can learn from their past mistakes and apply their skills in future practices. Before ascertaining the basketball score frequency and before determining the team strength between the players, it is important to collect the healthcare-related data of the players. The mental health-related determinants are more prominent in our research work as a team can perform well if they have cohesiveness and mental toughness to face all the situations in real-life traits. Hence, the study of complex health plays an important role in applying the algorithms to determine and evaluate the team strength in basketball players.

### 2.1. Variance Coefficient of Basketball Score Frequency

The score frequency is defined as the score divided by the time of playing. The score is usually used as a primary index to measure the quality of a team's scoring ability, i.e., the quality of the molecular system. However, there are some defects in using this primary index alone [8]. For example, A player gets 20 points in 40 minutes and B player gets 20 points in 20 minutes. Although A and B players have the same number of points, it is obvious that B player has more points in a unit time, and his scoring ability is considered better, however, the scoring index cannot reflect the players' advantages and disadvantages. To avoid the limitations of raw data, existing studies generally use a combination of hit ratios (hits/attempts, FGA%) to evaluate scoring ability [9].

From the statistical data, it is found that some players with weak scoring ability and less playing time rely on the extremely low number of trial shots to get a high hit rate. If player C only throws 2 baskets per game and hits 1 basket, then the FGA% is 50%. The hit rate has exceeded the average hit rate of NBA core scorers, however, it cannot be considered that the player has exceeded the core players in scoring ability. Therefore, the use of hit rate cannot be a good indicator to measure and evaluate the scoring ability of players [10]. To further measure and evaluate the scoring ability of players, it is necessary to reconstruct and optimize the primary index of scoring. It is considered that the index of score frequency is more scientific and accurate. Playing time itself can reflect a player's ability. Generally speaking, the coach will choose the players with a strong ability to play the game so that the players with high playing time may have a stronger ability. The higher scoring frequency depends on the higher number of scores, and the number of scores is highly related to the hit rate and shooting load, i.e., the higher number of scores requires the hit rate and the number of shots to be at a higher level. A higher hit rate and a higher number of shots mean that the player's scoring ability is stronger [11, 12].

### 2.2. Principle Model of Goal System for Basketball Players

In the process of setting up the principle model of the goal system of basketball players, the action point of the joint force when the ball is thrown is calculated, the action point of the joint force transmitted by the femoral head of the human body is shifted outward, the stress distribution curve of the femur under the action of the force on the femoral head is obtained, and the principal model of the goal system of basketball players is established [13, 14]. The specific steps are described as follows:

Assuming that *h*(*q*) represents the joint force transmitted by the femoral head in the process of pitching, *W*_*n*_ represents the gluteal muscle group's muscle force in pitching. *Z*^(*u*)^ represents the iliotibial band muscle force. The point of action of the joint force transmitted by the femoral head in pitching is calculated using the following formula:

(1) $$\begin{array}{c} Ρ\left(n\right)=\frac{Z^{\left(u\right)}\times h\left(q\right)}{W_{n}}\times \mu \left(F\right). \end{array}$$

In the formula, *μ*(*F*) is the thickness of the dense bone of basketball players.

Assuming that *s*(*i*) represents the thickness of the cancellous bone and *t*(*E*) represents the actual size of the human femur, formula (2) is used to offset the point of action of the joint force transmitted by the human femoral head when throwing the ball to obtain the stress distribution curve of the femur under the force of the femoral head.

(2) $$\begin{array}{c} \nu \left(\varepsilon \right)=\frac{t\left(E\right)\times s\left(i\right)}{g\left(E\right)}\times \frac{\lambda \left(P\right)\times \eta \left(Η\right)}{\mu \left(O\right)}\times Κ\left(S\right). \end{array}$$

In the formula, *g*(*E*) represents the sagittal axis in the coronal plane when pitching, *λ*(*P*) represents the abduction angle of the hip joint when pitching, meeting the condition of *p*=1,2,3 … *j*, *η*(Η) represents the continuous section of the upper femur when pitching, *μ*(*O*) represents the stress value of the posterior femoral neck when pitching, and *K*(*S*) represents the stress value of the posterior medial femur when pitching.

Assuming that *σ*′ represents the maximum abduction angle of the hip joint and *γ*(*p*) represents the variation of the stress values in the posteromedial and posteromedial parts of the femoral neck, the cross-sectional stress of the human joint is obtained by the following formula:

(3) $$\begin{array}{c} \kappa \left(e\right)=\frac{\sigma^{\prime }\times \nu \left(l\right)}{\Sigma \left(a\right)}\times \frac{E\left(Z\right)\times j_{o}+h_{j}}{\mu_{m}\times \gamma \left(p\right)}. \end{array}$$

In the formula, *ν*(*l*) represents the friction coefficient of the femur, Σ(*a*) represents the maximum influence function of different boundary conditions on the stress value, *E*(*Z*) represents the stress distribution of the femur under peak joint load, *j*_*o*_ represents the joint force transmitted by the femoral head, *o* represents the stress cloud value in the horizontal direction when ∂ is 0 mm, 5 mm, 10 mm, and 15 mm, *h*_*j*_ represents the stress value of human femoral neck under the combined load of bending and compression, and *μ*_*m*_ represents the cross-sectional stress of the upper end of the femoral shaft.

Assuming that *I*(*E*) represents the maximum stress of the femoral condyle during pitching, we use formula (4) as the principal model of the basketball players' pitching target system.

(4) $$\begin{array}{c} A\left(g\right)=\frac{I\left(E\right)\times \kappa \left(e\right)}{\phi \left(E\right)}\times R\left(w\right). \end{array}$$

In the formula, *ϕ*(*E*) represents the average width of the medullary cavity between the trabeculae, and *R*(*w*) represents the ratio of bone surface area to bone volume.

The correlation model of basketball shooting percentage is shown in Figure 1.

The analysis of stress and strain variation characteristics of basketball players in the process of pitching should be taken as the basis of training guidance. However, the traditional method completes the training by analyzing the biggest influencing factors of basketball players' goal skill training by different boundary conditions [15–17], but it cannot accurately analyze the stress and strain variation characteristics of the basketball players in the process of pitching. The result is that the training of pitching skills cannot achieve the effect [13, 18].

### 2.3. Team Strength Evaluation Algorithm under Cascade Feature Extraction

#### 2.3.1. Cascade Feature Extraction

Randomly select a basketball scoring video as the target of feature extraction, and finalize the Gabor filter transformation features. The four frequencies from eight directions are considered, and the direction value of *M* is presented as

(5) $$\begin{array}{c} M=\left(0,\frac{\pi }{8},\frac{2\pi }{8},\frac{3\pi }{8},\frac{4\pi }{8},\frac{5\pi }{8},\frac{6\pi }{8},\frac{7\pi }{8}\right). \end{array}$$

Under the above direction values, extract the characteristic values of the direction, respectively, set the basketball score image [19] after direction value processing to *I*(*x*, *y*), and the complex characteristic value of the moving image are given in the following equation:

(6) $$\begin{array}{c} g\left(x,y\right)=I\left(x,y\right)+\frac{\lambda^{2}+\gamma^{2}}{2\sigma^{2}}+\psi . \end{array}$$

In formula (6), *λ* represents the wavelength of sinusoidal function, *σ* represents the standard deviation of Gaussian function, *γ* represents the aspect ratio of space, and *ψ* indicates the phase shift. During cascade feature extraction, when cascading the above complex features, the real part and imaginary part of the complex features are filtered. The filtered complex features are given in the following equation:

(7) $$\begin{array}{c} \left\{\begin{array}{c} S=\cos\;i\left(2\pi \frac{\lambda }{\sigma }+\psi \right),\\ X=\sin\;i\left(2\pi \frac{\lambda }{\sigma }+\psi \right). \end{array}\right. \end{array}$$

In formula (7), *i* represents the direction of characteristic parameters, and the interpretation of other attributes remains unchanged. The real and imaginary portion of the composite features of the basketball scoring video image is used as the cascade object [20], and the cascade object is expressed in the following equation:

(8) $$\begin{array}{c} S_{tx}=\left[\begin{array}{cccc} S_{X_{1}}\left(1\right) & S_{X_{1}}\left(2\right) & \cdots & S_{X_{1}}\left(n\right)\\ S_{X_{2}}\left(1\right) & S_{X_{2}}\left(2\right) & \cdots & S_{X_{2}}\left(n\right)\\ \vdots & \vdots & \ddots & \vdots \\ S_{X_{n}}\left(1\right) & S_{X_{n}}\left(2\right) & \cdots & S_{X_{n}}\left(n\right) \end{array}\right]. \end{array}$$

In formula (8), *S*_*tx*_ indicates the cascaded set of composite features, and *n* indicates the dimension of the cascaded features. With the cascade set built by the above calculation formula, the cascade process shown in Figure 2 is constructed.

In Figure 2, the process begins with the feature extraction of basketball video, and the RGB color method is utilized to characterize the color elements in image [21]. The calculation formula is given in the following equation:

(9) $$\begin{array}{c} \left\{\begin{array}{c} R=\int_{\theta }E\left(\theta \right)S_{R}\left(\theta \right)d\theta ,\\ G=\int_{\theta }E\left(\theta \right)S_{G}\left(\theta \right)d\theta ,\\ B=\int_{\theta }E\left(\theta \right)S_{B}\left(\theta \right)d\theta . \end{array}\right. \end{array}$$

In formula (9), *S*_*R*_, *S*_*G*_, and *S*_*B*_, respectively, represent the filters of different colors, *E*(*θ*) represents light entering the filter, and *θ* represents the wavelength of light. Given the above calculation formula, an interval [0,1] forms an area to be detected, and the whole embedded basketball scoring video can be divided into three fan-shaped areas, and the area is given by the following equation:

(10) $$\begin{array}{c} A=r\frac{S\;\cos\;H}{2\;\cos\left(60^{\circ }-H\right)}. \end{array}$$

In formula (10), *A* represents the area, *r* represents the sector radius, and the meaning of other parameters remains unchanged. Using the real part and imaginary part of the complex feature of the basketball scoring video image as the cascade object, the color feature of the basketball scoring video is extracted to complete the target extraction of the cascade feature. The fan-shaped area composed of the above cascade features is used as the detection area to construct the basketball scoring frequency variation coefficient of the basketball scoring video.

#### 2.3.2. Basketball Scoring Video Target Detection

Taking the detection area composed of the above cascade features as the main detection object, the integral image value at any pixel in the sector area is defined, and the calculation formula can be expressed as

(11) $$\begin{array}{c} I_{i}\left(x,y\right)=\sum_{x^{\prime }\leq x,y^{\prime }\leq y}A\left(x^{\prime },y^{\prime }\right). \end{array}$$

In formula (11), *x*′ and *y*′ represent the coordinate values of any point in the detection area. To simplify the process of integrating the image value, the pixel points obtained by the above calculation formula are subtracted using the vertex integration diagram to control the calculation amount of integration. The subtraction process is shown in Figure 3.

According to the subtraction process shown in Figure 3, the basketball score frequency variation coefficient detection area is continuously cut to form a target detection area D. To ensure the accurate detection of the target detection area in the basketball scoring video playing process, a weighted superimposed strong classifier is used to construct a video conversion discrimination rule. The regularization formula can be expressed as

(12) $$\begin{array}{c} h_{j}\left(x\right)=\left\{\begin{array}{cc} 1 & \sum_{t=1}^{T}\alpha_{t}h_{t}\left(x\right)\geq \frac{1}{2}\sum_{t=1}^{T}\alpha_{t}\\ 0, & \text{otherwise} \end{array}|.\right. \end{array}$$

In formula (12), *h*_*t*_ represents the classifier feature, *α*_*t*_ represents the conversion threshold, and *T* is the frame rate of basketball scoring video. There are many detection factors in the variation coefficient of basketball scoring frequency. When the strong classifier is actually used, the too fast passing speed will lead to the delay of detection speed and cannot meet the requirements of target tracking. In the basketball scoring video image subwindow, a strong classifier cascade is constructed to identify the detection target. The cascade structure of strong classifiers is shown in Figure 4.

Under the control of the strong classifier cascade structure shown in Figure 4, scale the pixel ratio of the basketball score video to 20 ∗ 20 and enter the strong classifier cascade structure. The classifier determines the basketball score video area and rejects some images by the classifier. The rejected images will be input into the next classifier and is finally classified layer by layer. Complete the target detection of basketball score frequency variation coefficient and build the team strength evaluation algorithm based on this detection.

#### 2.3.3. Build Team Strength Evaluation Algorithm

When constructing the team strength evaluation algorithm, the classifier of basketball scoring video target detection is trained to form a detection and tracking process. The training process is expressed by the following equation:

(13) $$\begin{array}{c} G_{BN}={\sum_{i}\left(f\left(x_{i}\right)-y_{i}\right)}^{2}+\varepsilon {\left\|w\right\|}^{2}. \end{array}$$

In formula (13), *ε* represents the regularization parameter, *w* represents the number of classifiers, *f* represents the training function, *x*_*i*_ and *y*_*i*_ represent the independent and dependent variables of the function, and *i* represents the training times. To prevent fitting in the classifier training process, the optimal solution of the aforementioned calculation formula (13) is taken, and the calculation formula of the optimal solution can be expressed in the following equation:

(14) $$\begin{array}{c} w=\sum \alpha_{i}\varphi \left(x_{i}\right). \end{array}$$

In formula (14), *α*_*i*_ represents the coefficient of conversion solution, and *φ*(*x*_*i*_) represents the kernel function of training sample *x*_*i*_ mapped to high-dimensional space. The correlation between the 2 samples is determined as given in the following equation:

(15) $$\begin{array}{c} \varphi^{T}\left(x\right)\varphi \left(\dot{x}\right)=k\left(x,\dot{x}\right). \end{array}$$

In formula (15), *x* and $\dot{x}$, respectively, represent different samples, *k* represents Gaussian kernel function, and the value of conversion coefficient is deduced and calculated according to the functional relationship. The calculation formula can be expressed in the following equation:

(16) $$\begin{array}{c} \alpha ={\left(K+\lambda \delta \right)}^{-1}y. \end{array}$$

In formula (16), *K* represents the elements in the coefficient matrix, *δ* represents the identity matrix, and Fourier transform the above calculation formula (16) to obtain the following equation:

(17) $$\begin{array}{c} F\left(\alpha \right)=\frac{F\left(y\right)}{F\left(k^{xx}\right)+\lambda }. \end{array}$$

In formula (17), *F* represents the discrete Fourier transform and *k*^*xx*^ represents the first row vector of the kernel matrix, takes the optimal coefficient processed by the aforementioned calculation formula as the target template, takes the target template as the new input image *z* during actual target tracking, uses the Gaussian kernel to calculate the similarity between the input image and the target template, and constructs the basketball score video sample set. The processing matrix defining cyclic displacement is *K*^*z*^, which can be expressed in the following equation:

(18) $$\begin{array}{c} K^{z}=C\left(k^{xz}\right). \end{array}$$

In formula (18), *k*^*xz*^ represents the first row of the *K*^*z*^ matrix and *C* represents the cyclic movement coefficient of the matrix. The tracking process after the aforementioned calculation and processing is transformed into a diagonal matrix, and the product of the diagonal matrix and one-dimensional vector is transformed into point product operation, which realizes the target tracking and detection of the team strength evaluation algorithm. According to the particularity of the basketball score frequency variation coefficient, the histogram of the gradient direction amplitude value in the basketball score image unit is counted as the contour and shape information of the team strength evaluation target. By calculating the optimal solution of training basketball score video target detection classifier, the conversion coefficient value is deduced according to the function relationship. The Gaussian kernel is used to calculate the similarity between the input image and the target template to construct the basketball score video sample set, and the sequence results of the basketball score video are obtained. Based on the aforementioned calculation and processing, the construction of the team strength evaluation algorithm based on the basketball score frequency variation coefficient is finally completed.

## 3. Analysis of Experimental Results

To verify the effect and feasibility of the team strength evaluation algorithm based on the variation coefficient of basketball scoring frequency, an experimental analysis is carried out. The experiment uses MATLAB to design the algorithm. The resolution of the sampling of basketball score frequency variation coefficient is 600 × 800 pixels, and the template matching coefficient is 0.3. According to the aforementioned simulation environment and parameter settings, the team strength evaluation algorithm based on basketball score frequency variation coefficient is simulated.

The real game data of the 2017–2018 season provided by the NBA Database Chinese network is used as the experimental dataset of this paper, and the specific data content is shown in Table 1.

The integrated dataset is written into the HBase database, which makes the calculation more convenient. When HDFS reads and writes files, the program executes more quickly. The HBase database operation needs an HDFS file system as the bottom layer support, and the HBase database is the most basic storage unit of the HDFS file system in operation. At the same time, the programming mode of MapReduce operates the HBase database when implementing algorithms. Therefore, the HBase database is a bridge between the HDFS file system and MapReduce, which is a perfect combination of the three. A table created in the HBase database can be regarded as an infinite table. The fields of this table can be added and deleted dynamically according to the requirements. Column family and row key of the table must be declared when the table is defined. This flexible and fast feature of the table in the HBase database is very suitable for storing and studying the NBA team game data. In this paper, the map function operation process data in MapReduce exists in the form of key/value, while the table column family of the HBase database is a value and row key is the key.

According to the actual needs of the experiment, 30 data tables will be set up, which are the game information of NBA30 teams. The game data stored in these 30 tables will be programmed in the MapReduce module to realize the data involved in the sportrank algorithm and PageRank algorithm. The design content of team information table is shown in Table 2.

Table 2 team information table consists of one row key and three column families. Id represents the team ID, which is the row key of the table and the unique value. You can obtain information by querying the unique ID value. The column family with the field name results stores the team's victory or defeat. Result: 1 represents the winning rate and result: 0 represents the failure. Diff is the difference in the competition. Sr is the sportrank value, which is the strength value of the evaluation.

According to the relationship between NBA teams, from the perspective of the graph, it can be compared to a directed graph *G* (*U*, *R*). The node set *u* represents the team node set, and *R* represents the game relationship between the teams, as shown in Figure 5.

1. U: the node set composed of all teams, as shown in Figure 5, U = {Aa, Bb, Cc, Dd}.
2. R: by the competition between teams, a set of directed sides is formed R = {Aa⟶Bb，Aa⟶Cc，Aa⟶Dd，Bb⟶Aa，Bb⟶Dd，Dd⟶Bb，Dd⟶Cc}
3. Aa⟶Bb: it shows that the team aa loses to bb, the user Aa votes for bb, and calls Aa the follower of bb, and Bb the leader of aa.
4. Team's degree: the definition of out degree is the number of teams lost to other teams. For example, the team Aa's output is 3, and the user Bb's output is 2, which means that aa lost 3 games and bb lost 2 games.

According to the game relationship between the teams, the data model only needs to express the team's game situation to determine a complete relationship graph or adjacency matrix table as shown in Table 3.

The experimental dataset shown in Table 3 is used for experiments. The algorithms in reference [5], reference [6], and this paper are used to compare the performance of the three algorithms. Based on the aforementioned experimental preparation, take the team strength evaluation algorithm as the time record point and the computer evaluation box as the time statistical cut-off point and measure the running time of the 3 methods.  Figure 6 displays the results.

The evaluation execution time of the three methods rises as the number of datasets grows, according to the experimental results in Figure 6. The evaluation execution time of the algorithm in reference [5] is 8 s when the datasets reach 7, the evaluation execution time of the method in reference [6] is 11 s, and the evaluation execution time of the algorithm in this article is 4 s when the datasets reach 7. Therefore, it can be seen that the evaluation execution time of the algorithm in reference [6] is the longest, the evaluation execution time of the algorithm in reference [5] is the second, and the evaluation execution time of the algorithm in this paper is the shortest compared with the two algorithms, which has high timeliness.

Keep the experimental environment unchanged, take the number of frames in the experimental data set as the experimental object, and set the basketball scoring video. During the playback process, the team strength evaluation target has always been within the evaluation range, stipulating that the evaluation target can still be locked after the evaluation target is blocked as a successful evaluation process. Summarize and count the number of marker targets that can be evaluated by the three algorithms. The number of tag targets successfully evaluated is shown in Table 4.

According to the experimental results shown in Table 2 and Figure 7, the three algorithms show different team strength evaluation effects for the basketball score video data set prepared for the experiment. Taking the marked targets in the experimental preparation stage as the experimental object, the average number of successfully evaluated marked targets of the algorithm in reference [5] is about 14, and the number of successfully evaluated targets is the smallest. The average number of labeled targets successfully evaluated by the algorithm in reference [6] is about 23, which is more than that in reference [5]. However, the difference between the number of labeled targets and the algorithm in this paper is small, which can accurately evaluate the labeled targets of basketball video, and the evaluation effect is the best. To sum up, the team strength evaluation algorithm studied in this paper has the shortest execution time and more successful evaluation targets, which is more suitable for team strength evaluation based on basketball score frequency variation coefficient.

## 4. Discussion

### 4.1. Summary

A table is created in the database by the team strength evaluation algorithm based on the score frequency mutation coefficient. The table can be viewed as an infinite table whose fields can be dynamically added or deleted as required. The table's column family and row keys must be specified when the table is defined. The flexible and fast nature of tables in databases is ideal for storing data on NBA teams. Function operations have data in the form of keys/values, with the database's list family as the value and the row key as the key. The research on the team strength evaluation algorithm based on the coefficient of variation of basketball score frequency can improve the problems of the long execution time of the current team strength evaluation algorithm and the small number of successful evaluation marker targets, provide a theoretical research direction for the research of team strength evaluation algorithm, and meet the real-time needs of the coefficient of variation of basketball score frequency in team strength evaluation.

### 4.2. Prospects

It has a certain reference value for the competitive team strength evaluation method and specific algorithm implementation, however, because of the limitation of time and ability, there are still some deficiencies that need to be improved and perfected in the future research. Its deficiencies are mainly as follows:

1. Only after a match is over can the current group's strength be evaluated. If the group's strength is greatly reduced because of the injury or the absence or transaction of the players within the group, but the algorithm cannot be found in time, then it needs several more matches to evaluate the group's strength after the decline.
2. It is impossible to assess the strength of a team before any competition is held, and when there is little data on the team, the assessed strength of the team will be far from the actual strength. Only when the number of matches reaches a certain level can the accurate assessment be made.

### 4.3. Successful Target Achievements

The target achievement by the teams is an important parameter, and seven different datasets are used to check the viability of the proposed method. The target success is measured in percentage to check the accuracy of the healthcare-related data collected from the players and the dataset values that depict the change in the success rate of teams after devising our proposed algorithm. As per dataset 1, the accuracy is 86%, and the success rate for achieving the target is 97%. As per dataset 2, the accuracy is 87%, and the target achievement rate is 97.5%. As per dataset 3, the accuracy achieved is 89%, and the success rate achieved is 94.8%. The accuracy of results as per dataset 4 is 91%, and the target success rate achieved is 94.6%. The accuracy of dataset 5 is 93%, and the target success rate achieved is 94.5%. The accuracy of dataset 6 is 96%, and the target success rate achieved is 99.9%. The accuracy of dataset 7 is 96%, and the target success rate achieved is 98%.

## 5. Conclusions

The team's winning or defeating rate is not the only criterion to judge the strength of the team. There are many factors responsible in determining the strength of the team. Therefore, this paper has designed a team strength evaluation algorithm based on the variation coefficient of basketball scoring frequency. IoT and smart devices are used to collect data. The approach eliminates mistake accumulation, collects cascade characteristics from the basketball score video, creates video conversion discrimination rules, recognizes the basketball target, and obtains tracking target shape and frame information. Finally, it realizes the target tracking detection of the team based on the team strength using an evaluation algorithm. The evaluation of the team strength is made on the basis of the variation coefficient of basketball score frequency. The empirical results presented in the paper show that the designed algorithm has the shortest execution time, more successful evaluation targets between 94% and 97.6%, high efficiency with an accuracy of 97%, and more reliability in evaluating the strength of the team.

## Figures and Tables

**Figure 1:** Correlation model of basketball shooting percentage.

**Figure 2:** Characteristic cascade process.

**Figure 3:** Subtraction process.

**Figure 4:** Cascade structure of strong classifiers.

**Figure 5:** Team game relationships.

**Figure 6:** Evaluation execution time of different algorithms.

**Figure 7:** Marker targets evaluation chart depicting successfully completed targets.

**Table 1:** Basic information of teams.

ID	Team	Time	Opponent	Win or fail	Score	Opponents score	Absolute value of difference
1	Cleveland Cavaliers	2017.10.17	Boston Celtics	Win	102	99	3
2	Cleveland Cavaliers	2017.10.20	Milwaukee Bucks	Win	116	97	19
3	Cleveland Cavaliers	2017.10.21	Orlando Magic	Fail	93	114	21
4	Cleveland Cavaliers	2017.10.24	Chicago Bulls	Win	119	112	7
5	Cleveland Cavaliers	2017.10.25	Brooklyn Nets	Fail	107	112	5
6	Cleveland Cavaliers	2017.10.28	New Orleans Pelicans	Fail	101	123	22
7	Cleveland Cavaliers	2017.10.29	New York Knicks	Fail	95	114	19
8	Cleveland Cavaliers	2017.11.01	Indiana Pacers	Fail	107	124	17
9	Cleveland Cavaliers	2017.11.03	Washington Wizards	Win	130	122	8
10	Cleveland Cavaliers	2017.11.05	Atlanta Hawks	Fail	115	117	2
…	…	…	…	…	…	…	…

**Table 2:** Design of team information table.

Line key	Lie clan			
	Result	Opponent	Diff	SR
Id:1	Result:1 Result:1 Result:0 Result:1 …	Opponent:1 Opponent:5 Opponent:17 Opponent:4 …	Diff:3 Diff:18 Diff:21 Diff:7 …	SR:1 SR:21 SR:13 SR:2 …

**Table 3:** Adjacency matrix table.

Team ID	Leader's ID
Aa	Bb, Cc, Dd
Bb	Aa, Dd
Cc	Cc
Dd	Bb, Cc

**Table 4:** Number of marker targets successfully evaluated by different algorithms.

Data set serial number	Number of tracking targets/piece			
	Mark target	Reference [5] algorithm	Reference [6] algorithm	Paper algorithm
1	44	13	23	43
2	41	14	22	40
3	39	11	24	37
4	38	10	23	36
5	37	16	23	35
6	30	15	20	30
7	36	18	27	35

## Data Availability

Data will be made available on request from the author.
